This article has been retracted.

# Effect of Yifei-Huoxue Decoction Combined with Tiotropium on Inflammatory Cytokine Levels, Pulmonary Function, and Quality of Life in Patients with Chronic Obstructive Pulmonary Disease

**DOI:** 10.1155/2022/5740181

**Published:** 2022-05-19

**Authors:** Yunjiao Sheng, Yang Li, Ting Feng

**Affiliations:** ^1^Department of Health Care, Jinan Municipal Hospital of Traditional Chinese Medicine, Jinan 250000, Shandong, China; ^2^Department of Pharmacy, Qingdao Municipal Hospital, Qingdao, China; ^3^Department of Pulmonary Disease, Jinan Municipal Hospital of Traditional Chinese Medicine, Jinan 250002, Shandong, China

## Abstract

**Objective:**

The main objective is to investigate the effect of Yifei-Huoxue decoction combined with tiotropium on the inflammatory cytokine levels, pulmonary function, and quality of life in patients with chronic obstructive pulmonary disease (COPD).

**Methods:**

Ninety-eight COPD patients who were treated in our hospital from January 2021 to January 2022 were selected as the research objects, and they were divided into reference group (routine treatment) and study group (Yifei-Huoxue decoction combined with tiotropium), with 49 cases in each group. The patients' clinical indexes were compared between the two groups, and the clinical efficacy in the two groups was analyzed.

**Results:**

Compared with the reference group, the study group had remarkably lower inflammatory cytokine levels (including tumor necrosis factor-*α* (TNF-*α*), C-reactive protein (CRP), and interleukin-6 (IL-6)) after treatment (*P* > 0.05). In terms of the patients' pulmonary function indexes after treatment, the study group achieved lower forced vital capacity (FVC), forced expiratory volume in 1s (FEV1), and FEV1/FVC levels compared with the reference group (*P* < 0.05). Both groups had a lower erythrocyte sedimentation rate (ESR) after treatment compared with that before treatment. However, the intergroup difference in the ESRs after treatment was remarkable, and the study group had a much lower ESR compared with the reference group (*P* < 0.05). Compared with the reference group, the study group achieved much higher 36-item short form health survey (SF-36) scores in dimensions of general health, physical functioning, social functioning, and mental health after treatment (*P* < 0.05).

**Conclusion:**

Yifei-Huoxue decoction combined with tiotropium not only enhances the COPD patients' pulmonary function but also decreases their inflammatory levels. Therefore, this treatment is conducive to promoting the COPD patients' recovery and exerts positive effect on improving their quality of life.

## 1. Introduction

Chronic obstructive pulmonary disease (COPD), as a chronic disease with restricted pulmonary airflow and irreversible and continuous respiratory dysfunction, is an intractable disease in the clinic. COPD has become a major chronic disease with a significant degree equivalent to diabetes and hypertension. According to the data released by the World Health Organization (WHO), COPD will be the 5th disease burden worldwide in 2022, which causes a huge disease burden on the physical health of humans. In recent years, traditional Chinese medicine (TCM) presents special advantages in treating COPD, and various research findings have shown the TCM characteristics of “mastering the initiative of life from breathing” [1–4]. Currently, the holistic thinking is mostly advocated in treating COPD in the clinic. In the acute phase of COPD, Western medicine generally adopts antibiotics, but the objects of antibiotic treatment are mainly the patients with a bacterial infection. For patients with virus infection, TCM is more effective. In addition, previous studies have shown that TCM, with satisfactory efficacy, can be applied in the whole course, no matter whether the patients with COPD are in the acute exacerbation phase or in the stable phase [5,6]. The acute exacerbation of the patients' conditions is an important cause of COPD progression and even death. Modern medicine takes antiinfection, resolving phlegm, and relieving cough and asthma as the main treatment principles, but the bacterial resistance to antibiotics and airway mucus hypersecretion are the main bottlenecks of Western medical treatment. According to the investigations [7,8], about 75% of patients at the acute stage of COPD belong to phlegm-heat obstructing lung, so taking Chinese medicine on the basis of Western medical treatment is more effective in shortening the course of the disease and promoting recovery. Standardized treatment and scientific management during the stable phase, effectively reducing the frequency of acute attacks and improving patients' quality of life, are important to prevent disease progression. A bronchodilator agent is the cornerstone of treatment during the stable phase. Tiotropium, an anticholinergic bronchodilator, is commonly used for the maintenance treatment of COPD in the clinic and has remarkable efficacy. The studies on the compound Chinese prescription during the stable phase mainly focus on the prescriptions for tonifying the lung, nourishing the spleen and kidney, activating blood, removing stasis, and expelling phlegm. The study of Kaiwen et al. [9], by revealing the mechanism of the compound TCM's intervention on airway mucus hypersecretion, airway remodeling, and oxidation-antioxidant imbalance from multiple perspectives, provides strong theoretical support for the TCM treatment for COPD. Based on this, this paper investigates the clinical efficacy of Yifei-Huoxue decoction combined with tiotropium in treating COPD, so as to provide new thoughts for the clinical treatment of this disease.

## 2. Materials and Methods

### 2.1. Inclusion and Exclusion Criteria

According to the research object, the inclusion criteria were set as follows: ① the patients met the diagnostic criteria of COPD in *GOLD Global Strategy for the Diagnosis, Management, and Prevention of Chronic Obstructive Pulmonary Disease (2021)* [10] and *diagnostic criteria of TCM Syndromes in Chronic Obstructive Pulmonary Disease (2011)* [11]; ② the patients were in stable period; ③ according to the severity of COPD graded by FEV1/FVC, patients with an FEV1/FVC level of 30–70% were included, and the very severe patients were excluded; ④ the patients had no contraindication for tiotropium, and they were over 18 years old; ⑤ the patients and their families were informed of this study and signed the informed consent. Exclusion criteria were set as follows: ① the patients had a history of taking glucocorticoids and bronchodilator agents for a long time; ② the patients' pulmonary disease was caused by pulmonary tuberculosis, tumor, bronchial dilation, and other factors; ③ the patients were complicated with severe and unstable organic dysfunction; ④ the patients' treatment compliance was poor or their clinical data were incomplete; ⑤ the patients could not state their chief complaint clearly.

### 2.2. Screening and Grouping

According to the above criteria, 98 COPD patients who were treated in our hospital from January 2021 to January 2022 were selected as the research objects, and a retrospective study on these patients was conducted. According to the therapeutic regimens the patients received, they were divided into the reference group (routine treatment) and study group (Yifei-Huoxue decoction combined with tiotropium on the basis of routine treatment), with 49 cases in each group. This study met the World Medical Association Declaration of Helsinki (2013) [12].

### 2.3. Treatment Methods

The reference group received routine treatment, namely symptomatic treatment. According to the clinical treatment experiences and the patients' case history, the patients were given antibacterial agents, oxygen inhalation with low volume (the respirator was adopted to support respiration when necessary), and expectorants. In addition, nondrug therapies were also conducted, such as persuading the patients into quitting smoking, and for those with COPD due to dust, irritant gas, or their occupations, occupational protection was enhanced, and regular physical examination should be done.

The study group received Yifei-Huoxue decoction combined with tiotropium on the basis of routine treatment. ① Tiotropium bromide powder for inhalation (Manufacturer: Xianju Pharmaceutical Co., Ltd., NMPA approval no. H20090279, specification: 18 *μ*g/*a* capsule) was used. When using, one capsule was put into the piercing slot of a special aspirator, and the button was pressed by the finger. Both ends of the capsule were punctured by a fine needle, and then, the oral aspirator was put into the deep part of the oral cavity. Then, the patients inhaled with an effort, and the capsule rotated rapidly with the airflow. Following that, the powder in the capsule was sprayed out of the capsule shell and entered the respiratory tract with the airflow. The patients took one capsule each time and once a day. ② Yifei-Huoxue decoction. The components of this decoction were 24g of rehmannia glutinosa, 18g of dwarf lilyturf root, 15g of dangshen, 15g of membranous milkvetch root, 15g of the root of straight ladybell, 15g of twotooth achyranthes root, 12g of chuanxiong rhizome, 12g of largehead atractylodes rhizome, 12g of Chinese angelica root, 9g of safflower, 9g of peach seed, 9g of balloon flower root, and 6g of licorice. The above medicinal herbs were decocted with water, and one potion was 500 ml. The patients took one potion a day and took the warm decoction twice a day in the morning and afternoon. The treatment cycles in both groups were 4 weeks.

### 2.4. Observed Indexes

General data. The patients' age, body mass index (BMI), course of the disease, sex, smoking, drinking, education level, place of residence, and other general data were analyzed and compared between the two groups.

Inflammatory cytokines. Five milliliters of fasting venous blood were drawn and collected from each patient. Then, the enzyme-linked immunosorbent assay was adopted to determine the patients' tumor necrosis factor-*α* (TNF-*α*), C-reactive protein (CRP), and interleukin-6 (IL-6) levels.

Pulmonary function. Before and after treatment, the spirometer (Model: master screen; Manufacturer: Germany Jaeger) was adopted to determine the patients' pulmonary function indexes, and the indexes included forced vital capacity (FVC), forced expiratory volume in 1s (FEV1), and FEV1/FVC levels. FEV1/FVC ≥70% indicated normal pulmonary function.

Erythrocyte sedimentation rate (ESR). The patients' fasting venous blood was drawn and collected in the morning to determine their ESR in the clinical laboratory of our hospital. The normal reference values of ESR for male and female were, respectively, 0–15 mm/h and 0–20 mm/h.

Quality of life. The 36-item short form health survey (SF-36) [13] was adopted to evaluate the patients' health, which was developed by the Boston Health Research Institute in the United States and has been widely used in the areas of quality of life measurement in the general population, evaluation of the effects of clinical trials, and health policy assessment. The modified scale mainly included four dimensions of general health, physical functioning, social functioning, and mental health. Higher scores indicated better quality of life.

### 2.5. Statistical Treatment

The statistical software SPSS22.0 was adopted to calculate intergroup differences, and GraphPad Prism 7 (GraphPad Software, San Diego, USA) was used to draw graphs of the data in this study. The research data included count data and measurement data, which were expressed by (n(%)) and (‾*x* ± *s*), respectively, and tested by X^2^ and *t*. When *P* < 0.05, the differences were considered statistically significant.

## 3. Results

### 3.1. General Data

No statistical difference in the patients' age, BMI, course of disease, sex, smoking, drinking, education level, place of residence, and other general data was observed between the two groups (*P* < 0.05; Table 1).

### 3.2. Inflammatory Cytokines

Compared with the reference group, the study group had much lower inflammatory cytokine levels (including TNF-*α*, CRP, and IL-6) after treatment (*P* < 0.05; Table 2).

### 3.3. Pulmonary Function

In terms of the patients' pulmonary function indexes after treatment, the study group achieved lower FVC, FEV1, and FEV1/FVC levels compared with the reference group (*P* < 0.05; Table 3).

### 3.4. ESR Levels

Both groups had lower ESR after treatment compared with that before treatment. However, the intergroup difference in ESR after treatment was remarkable, and the study group had much lower ESR compared with the reference group (*P* < 0.05; Table 4).

### 3.5. Quality of Life

Compared with the reference group, the study group achieved much higher SF-36 scores in dimensions of general health, physical functioning, social functioning, and mental health after treatment (*P* < 0.05; Figure 1).

Note: the abscissa represented evaluation dimensions, and the ordinate represented the score.

After treatment, the reference group's SF-36 scores in dimensions of general health, physical functioning, social functioning, and mental health were (5.72 ± 1.30), (5.54 ± 1.16), (5.97 ± 1.28), and (5.06 ± 1.10), respectively.

After treatment, the study group's SF-36 scores in dimensions of general health, physical functioning, social functioning, and mental health were (7.75 ± 1.36), (7.25 ± 1.02), (7.11 ± 1.27), and (6.35 ± 1.24), respectively.

*∗* represented the differences in patients' general health, physical functioning, social functioning, and mental health between the two groups after treatment (*t* = 7.553, 7.749, 4.426, and 5.448, *P* < 0.001).

## 4. Discussion

COPD is a common and frequently encountered respiratory disease and presents progressive development due to airflow limitation. COPD, with slow onset and long duration, seriously affects patients' labor ability and quality of life and brings a huge social and economic burden for the patients with the progressive decline of pulmonary function [14–16]. COPD is irreversible, and the main treatment principles are controlling disease development, enhancing lung function, and improving quality of life. Tiotropium, a novel bronchodilator and a long-acting anticholinergic agent, is suitable for the maintenance treatment of COPD and the prevention of acute attack. From the perspective of pharmacological action, tiotropium is a quaternary ammonium derivative and an anticholinergic agent with high selectivity. Tiotropium has the same affinity with the five types of M1-M5 muscarinic receptors and has a higher affinity with the receptors in the human airway. Besides, the dissociation of tiotropium with M1 and M3 muscarinic receptors is slow, and tiotropium can block the tracheobronchial smooth muscle contraction mediated by cholinergic nerves for a long time, showing a unique kinetic selectivity on M1 and M3 receptors. In addition, the dilating effect of tiotropium on bronchus can last for more than 24 hours, and the plasma concentration is about 2pg/ml, which presents that tiotropium has a long duration of action and is suitable for the long-term treatment of COPD in the stable stage. Therefore, tiotropium is conducive to protecting lung function, reducing the seizure frequency, and improving the patients' quality of life.

According to TCM, COPD belongs to the categories of “pulmonary distention” and “dyspnea”, and deficiency, phlegm, and stasis exist in the body through the progression of COPD. The deficiency of vital energy is the pathologic base of the occurrence and development of COPD. The deficiency of vital energy, initially originating from lung and spleen deficiency, gradually develops into the deficiency of lung, spleen, and kidney, damages yang qi, and causes asthenia of both yin and yang. Yin deficiency, mostly originating from lung-yin deficiency or lung and kidney yin deficiency, gradually develops into hepatic and renal yin deficiency and may damage some yang qi [17, 18]. “Phlegm turbidity and blood stasis” are not only the pathological products of the deficient internal organs but also the main pathogenic factors in the evolution of COPD. Deficiency in origin and excess in superficiality interrelate and deteriorate the disease, so the disease always recurs and the patients do not recover. As a result, the phlegm and blood are blocked in the pulmonary vessels. Therefore, the clinical syndrome differentiation should be conducted on the basis of qi, blood, yin, yang, and the deficiency syndrome of five viscera. Yifei-Huoxue decoction is developed by our hospital based on the previous research results, and it is composed of rehmannia glutinosa, dwarf lilyturf root, dangshen, membranous milkvetch root, root of straight ladybell, twotooth achyranthes root, chuanxiong rhizome, largehead atractylodes rhizome, Chinese angelica root, safflower, peach seed, balloonflower root, and licorice. In this decoction, dangshen, largehead atractylodes rhizome, and membranous milkvetch root can invigorate the spleen, excrete dampness, and resolve phlegm. Dangshen and membranous milkvetch root can also improve the transformation ability of lymphocytes and the phagocytic capacity of macrophages, and the combination of both can effectively enhance the patients' cell and humoral immunity, conducive to reducing blood viscosity, improving microcirculation, activating blood circulation, and dispersing stasis. Chinese angelica root, warm in nature, can activate blood circulation and replenish blood. The combination of Chinese angelica root and membranous milkvetch root has a better effect on improving blood circulation and can disperse stasis without causing blood disorder [19,20]. Besides, rehmannia glutinosa can remove heat to cool blood, promote fluid production, and invigorate yin. Dwarf lilyturf root, acting on heart, lung, and stomach meridians, can moisten the lung and clear away heart fire and has the function of reducing blood glucose and enhancing immunity and antibiosis. It is fair to say that dwarf lilyturf root is a good drug to invigorate yin and moisten the lung. The combination of dwarf lilyturf root and the root of straight ladybell, with a sweet flavour and cold nature, can promote the production of body fluid and nourish the lung and stomach. Chuanxiong rhizome, as a blood-activating and pain-alleviating drug subordinated to blood-activating and stasis-resolving drugs, has the function of regulating qi and dispelling wind evil. Peach seed can activate blood activation, disperse blood stasis, and relieve cough and asthma. Safflower can improve blood circulation to promote menstruation flow. The combination of balloonflower root and licorice can release pulmonary qi, relieve sore throat, invigorate spleen, and replenish qi. Twotooth achyranthes root can tonify the liver and kidney and enhance body immunity [21]. The combination of various herbs can complement each other in the treatment and exerts the functions of activating blood flow, removing blood stasis, strengthening the spleen, tonifying the lung, drying dampness, and resolving phlegm, so as to improve the nutrition and endurance of respiratory muscle, relieve the respiratory muscle fatigue, and enhance pulmonary function. A large number of previous clinical studies have shown that the bacterial resistance to antibiotics and airway mucus hypersecretion are the main bottlenecks of Western medicine in the treatment of acute and exacerbated COPD. The syndrome investigation with a large sample size has found that 75% of patients belong to the category of the phlegm-heat obstructing lung [22–24]. The TCM prescription formulated according to the symptoms has revealed the mechanisms from the aspects of reducing drug resistance, lowering airway mucus secretion, and enhancing anti-inflammatory effect, and the synergistic effect of TCM prescription with Western medical treatment has been confirmed. Based on this, the study has retrospectively analyzed the clinical data of some COPD patients treated in our hospital and investigated the efficacy of Yifei-Huoxue decoction combined with tiotropium in treating COPD.

According to the study results and the analysis of TNF-*α*, CRP, and IL-6, both groups had lower inflammatory cytokine levels after treatment compared with those before treatment, and the study group had markably lower inflammatory cytokine levels compared with the reference group (*P* < 0.05). The above study result conforms to the report of Dave et al [25]. Besides, both groups had lower ESR after treatment compared with that before treatment, but the intergroup difference in ESR after treatment was remarkable, and the study group had much lower ESR compared with the reference group (*P* < 0.05) At present, some studies have confirmed that the combination of CRP and ESR has effective value for predicting COPD patients' conditions and prognoses, so CRP level and ESR can reflect the patients' treatment situation. Hence, this study result has confirmed that Yifei-Huoxue decoction combined with tiotropium can effectively mitigate COPD patients' inflammatory response and improve the clinical efficacy. The pulmonary function test showed that the study group achieved lower pulmonary function indexes compared with the reference group (*P* < 0.05). The gold standard in clinical diagnosis of COPD is FEV1/FVC lower than 70%. According to the study results, the average value of FEV1/FVC in the reference group was 60.82% and in the study group was 74.10%, and the FEV1/FVC value in the study group was remarkably better than that in the reference group, indicating that Yifei-Huoxue decoction combined with tiotropium can effectively improve COPD patients' pulmonary function and accelerate their recovery. In terms of the patients' quality of life, the study group achieved much higher SF-36 scores in dimensions of general health, physical functioning, social functioning, and mental health after treatment compared with the reference group (*P* < 0.05), indicating that Yifei-Huoxue decoction combined with tiotropium further enhances COPD patients' quality of life. In the treatment of COPD, Yifei-Huoxue decoction does not stick to a certain method or herb, and the valuable point of syndrome differentiation and treatment lies in “grasping mechanism flex method”. Tiotropium, with high affinity with lung tissues, can antagonize free radicals and eliminate the damage of peroxides to lung tissues, so as to decrease the inflammatory reaction. This study has the following deficiencies. (1) This is a retrospective study based on the authors' clinical experiences and practical results. In this study, the sample size is small, and prospective studies with large sample size are needed to confirm the universality of Yifei-Huoxue decoction combined with tiotropium in the treatment of COPD; (2) COPD is a respiratory infectious disease, and the long efficacy of Yifei-Huoxue decoction and tiotropium on treating COPD is needed to be continuously investigated and verified in practice.

In conclusion, Yifei-Huoxue decoction combined with tiotropium not only effectively enhances the COPD patients' pulmonary function but also decreases their inflammatory levels. Therefore, this treatment is conducive to promoting patient recovery, has potential utility in the improvement of COPD patients' prognosis and quality of life, and provides a new medication idea for the clinical treatment of COPD.

## Figures and Tables

**Figure 1:** Patients' SF-36 scores.

**Table 1:** Comparison of the general data (*n* = 49).

Observed indexes	Reference group	Study group	X^2^/*t*	*P*
Age (years old)	64.72 ± 6.08	65.13 ± 6.15	0.332	0.741
BMI (kg/m^2^)	23.12 ± 3.01	23.24 ± 2.85	0.203	0.840
Course of disease (years)	9.05 ± 3.26	9.17 ± 3.15	0.185	0.853
Sex				
Male	29 (59.18)	31 (63.27)	0.172	0.678
Female	20 (40.82)	18 (36.73)		
Smoker	23 (46.94)	22 (44.90)	0.041	0.839
Drinker	25 (51.02)	24 (48.98)	0.041	0.840
Education level				
Under junior high school	21 (42.86)	19 (38.78)	0.169	0.681
Junior high school	16 (32.65)	17 (34.69)	0.046	0.831
Above junior high school	12 (24.49)	13 (26.53)	0.054	0.817
Place of residence				
Urban areas	31 (63.27)	33 (67.35)	0.180	0.671
Rural areas	18 (36.73)	16 (32.65)		

**Table 2:** Patients' inflammatory cytokine levels.

Observed indexes		Reference group (*n* = 49)	Study group (*n* = 49)	*t*	*P*
TNF-*α* (ng/L)	Before treatment	34.22 ± 3.17	34.56 ± 3.20	0.528	0.599
	After treatment	29.45 ± 2.17	25.94 ± 2.15	8.043	<0.001

CRP (mg/L)	Before treatment	7.12 ± 0.85	7.10 ± 0.84	0.117	0.907
	After treatment	4.88 ± 0.52	3.46 ± 0.51	13.647	<0.001

IL-6 (ng/L)	Before treatment	70.85 ± 4.73	70.52 ± 4.52	0.353	0.725
	After treatment	51.06 ± 3.34	26.75 ± 3.29	36.291	<0.001

**Table 3:** Patients' pulmonary function indexes.

Observed indexes		Reference group (*n* = 49)	Study group (*n* = 49)	*t*	*P*
FVC (L)	Before treatment	2.16 ± 0.22	2.14 ± 0.20	0.471	0.639
	After treatment	2.50 ± 0.21	2.75 ± 0.24	5.488	<0.001

FEV1 (L)	Before treatment	1.26 ± 0.29	1.25 ± 0.31	0.165	0.869
	After treatment	1.55 ± 0.34	1.86 ± 0.32	4.678	<0.001

FEV1/FVC (%)	Before treatment	55.33 ± 4.62	55.51 ± 4.58	0.194	0.847
	After treatment	60.82 ± 5.11	74.10 ± 5.20	12.751	<0.001

**Table 4:** Patients' ESR levels (mm/h).

Group	*n*	Before treatment	After treatment
Reference group	49	78.83 ± 7.25	60.17 ± 6.79
Study group	49	78.49 ± 7.17	37.65 ± 6.92
*t*		0.233	16.267
*P*		0.816	<0.001

## Data Availability

The data to support the findings of this study are available on reasonable request from the corresponding author.
